The article "Sparrow Search Algorithm-Optimized Long Short-Term Memory Model for Stock Trend Prediction" was published in 2022. Journal: Comput Intell Neurosci.

# Sparrow Search Algorithm-Optimized Long Short-Term Memory Model for Stock Trend Prediction

**DOI:** 10.1155/2022/3680419

**Published:** 2022-08-12

**Authors:** Feiyang Liu, Panke Qin, Junru You, Yanyan Fu

**Affiliations:** School of Software, Henan Polytechnic University, 454003 Jiaozuo, China

## Abstract

The long short-term memory (LSTM) network is especially suitable for dealing with time series-related problems, which has led to a wide range of applications in analyzing stock market quotations and predicting future price trends. However, the selection of hyperparameters in LSTM networks was often based on subjective experience and existing research. The inability to determine the optimal values of the parameters results in a reduced generalization capability of the model. Therefore, we proposed a sparrow search algorithm-optimized LSTM (SSA-LSTM) model for stock trend prediction. The SSA was used to find the optimal hyperparameters of the LSTM model to adapt the features of the data to the structure of the model, so as to construct a highly accurate stock trend prediction model. With the Shanghai Composite Index stock data in the last decade, the mean absolute percentage error, root mean square error, mean absolute error, and coefficient of determination between stock prices predicted by the SSA-LSTM method and actual prices are 0.0093, 41.9505, 30.5300, and 0.9754. The result indicates that the proposed model possesses higher forecasting precision than other traditional stock forecasting methods and enhances the interpretability of the network model structure and parameters.

## 1. Introduction

The financial market has social functions such as promoting economic development and optimizing resource distribution. Among them, the stock market has more lucrative investment returns than other fields. Investors need to grasp the changes in the stock market and accurately predict stock price trends to obtain considerable profits and avoid potential risks. Due to the constant development of financial markets and the intense demand from investors, stock price forecasting has attracted widespread attention in academic and business fields [1]. Stock prices are influenced by many factors and have many features such as high noise, and being dynamic, nonlinear, and nonparametric [2]. These factors make the research of stock price prediction to be a difficult task.

The traditional approach to stock forecasting is to analyze statistical and techno-charts and combine them with the experience of the investor. Some scholars arranged the daily prices of stocks in chronological order and built time-series models, such as the autoregressive integrated moving average (ARIMA) model [3]. This type of mathematical model is difficult to reach a high prediction accuracy due to the complex factors that affect stock prices.

With the growth of artificial intelligence and the age of big data, numerous researchers have started to focus on the massive data in the stock market. A growing number of studies are using artificial intelligence techniques for stock price prediction, and various stock prediction models have also been proposed [4]. Machine-learning methods such as support vector machines (SVM) have shown many advantages over traditional fundamental and technical analysis of the stock market, particularly in breaking through many of the limitations of traditional methods when dealing with large amounts of complex data. Deep learning has evolved at a remarkable pace over the last few years and has made significant breakthroughs in several fields. Research by many scholars has shown that deep learning models have more powerful feature extraction and generalization capabilities [5]. The long short-term memory (LSTM) network overcomes the problem of vanishing gradients, so it can effectively learn long-term dependencies through memory units, and the effect of the LSTM method is better than that of memoryless classification methods [6] and traditional recurrent neural network (RNN) [7]. Therefore, LSTM is more widely used when dealing with time-series data such as stock prices.

Although LSTM is a potent tool for time-series problems, it still has some shortcomings. First, network models such as LSTM lack the ability to explain the final decision-making obtained by the model and to provide a specific explanation of the parameters used to achieve the prediction results [8]; and second, the setting of hyperparameters in the model is often based on existing research or experience and has a certain degree of subjectivity. Appropriate hyperparameters can improve the topology of the network model and enhance the generalization and fitting abilities. Therefore, how to eliminate the influence of human factors and find the optimal network hyperparameters is also a research concern for scholars.

Given the above problems, we use the sparrow search algorithm [9] for optimizing LSTM networks and propose an SSA-LSTM stock trend prediction model. A new population intelligence optimization algorithm was applied in this study to discover the optimal values of the parameters of the LSTM network. This process provides an answer to the problem that LSTM cannot explain how the model gets the ability to make final decisions and is subject to human factors. We use a dataset of Shanghai Composite Index stocks in the Chinese market from 2010 to 2021 for empirical analysis. The contribution of this research can be described in two points:

1. This paper designed an LSTM model optimized by the SSA to forecast stock price trends.
2. To verify the effectiveness of the sparrow search algorithm-optimized LSTM (SSA-LSTM) model, we perform comparative experiments using back-propagation (BP) neural network models, RNN models, LSTM models, gated recursive unit (GRU) models, and the particle swarm optimization algorithm-optimized LSTM (PSO-LSTM) model. The results prove that SSA-LSTM has the performance of tracking the stock price trend, and the prediction accuracy is superior to other methods.

The remaining chapters of this article are organized as follows: The second part is the related work, which mainly analyzes the research status in the field of stock forecasting and the application of LSTM in this field; the third part introduces the SSA-LSTM model; the fourth part is the experimental results of the SSA-LSTM and other models for stock price prediction; and the last part is the conclusion of this work.

## 2. Related Works

Kim [10] used the SVM to predict the Korea Composite Stock Price Index. The results of the experiments demonstrated that this method is more effective than the traditional neural network method. Wang [11] used BP neural network and improved it. The analysis shows that the model is feasible and effective, with increased forecast precision compared with that of the original BP network. Ticknor [12] fed daily market prices and company financial indicators into a feed-forward neural network model to predict the stock prices of Microsoft and Goldman Sachs. Jia et al. [13] proposed a segmented gray-autoregressive moving average (ARMA) model recursive algorithm and a segmented artificial neural network (ANN)-ARMA recursive algorithm based on the idea of wavelet decomposition reconstruction. After the process of decomposition modeling and reconstruction, both of these models showed satisfactory prediction accuracy in short-term forecasting. Rather et al. [14] combined the RNN, ARMA, and exponential smoothing models to form a new regression model. It overcomes the limitations of linear models and achieves satisfactory prediction results.

Lv et al. [15] designed a LightGBM-optimized LSTM model to combine multitask learning with LSTM networks for stock market forecasting. Zheng et al. [16] used a series of uniformly distributed random data based on an LSTM model to predict stock market indices. Gao et al. [17] innovatively integrated multiple technical indicators, including financial data, to compare the stock market prediction performance between LSTM and GRU under different parameters. Wang et al. [18] proposed a convolutional neural network (CNN)-bidirectional special long short-term memory (BiSLSTM) composite model to predict the closing price of stocks in the coming day. The CNN is in charge of capturing the characteristics of the input data in this model, and the bidirectional long short-term memory (BiLSTM) is employed to consider the changing patterns of the historical data. With further studies of stock prediction, researchers have found that various auxiliary indicators play a critical role in stock price prediction. Fu et al. [19] proposed an LSTM stock trend prediction model that fuses multisource information. The method introduces technical stock indicators and financial text features in addition to the basic stock data features. The experimental results demonstrate that both economic text features and stock technical indicators have a positive impact on improving the predictive capacity of the model. In another recent work, Li et al. [20] proposed a prediction model based on multiview features. The method applies different stock technical indicators as features from different perspectives and uses LSTM and deep neural networks to develop an ensemble learning prediction model. The final experiment proves that the model not only performs well in predicting U.S. news stock prices but also can analyze the effects of different stock technical indicators on the prediction results.

In 2018, Chung and Shin [21] applied genetic algorithms to find the optimal values of time step and number of neurons in the LSTM network model. They selected the Korean Stock Price Index for testing and proved that the optimized model outperformed the benchmark model. In 2019, Song et al. [22] optimized the time step, the batch size, the number of iterations, and the number of hidden layer neurons in LSTM networks using the particle swarm optimization algorithm with an adaptive learning strategy. The experiment results of predicting the stock market in Shanghai and Shenzhen demonstrate that the optimized LSTM has certain universality and good prediction accuracy. Researchers such as Hu [23] optimized the learning rate, the number of hidden layers, and the number of neurons of LSTM through a Bayesian algorithm to predict the stock prices of leading stocks at specific stages of the Chinese stock market. The experimental results demonstrate that the optimized model has high generality and efficiency. Liao [24] applied the sparrow search algorithm to optimize the weights, bias, the number of neurons in the hidden layer, and the number of iterations of the LSTM network. This approach has improved the prediction accuracy of the model and has been successfully applied to load forecasting problems with good results.

## 3. Methodology

### 3.1. Sparrow Search Algorithm

The SSA is a novel group intelligence optimization algorithm influenced by the foraging process of sparrows. The sparrow foraging process is a kind of producer-scrounger model with an investigation mechanism and an early warning mechanism. Producers have a high value of fitness. Producers are in charge of seeking food, offering foraging areas, and providing movement directions for scavengers. Scavengers increase their fitness value by following producers who own the optimal fitness value to gain food. In addition, some scroungers will monitor the energy status of the producers. A part of the scavengers will actively snatch food if the producer has a high energy level. Once the sparrow finds a predator, it will immediately send an alarm signal and move to a safe area. In the central part of the population, sparrows move randomly toward their companions. Producers need to lead scroungers out of the danger zone when the safety threshold is lower than the alarm value.

Assuming that the sparrow population is *n* and in a *d*-dimensional search area, the location information of each individual can be regarded as an *n* × *d*-dimensional matrix at this time. The position of each sparrow can be presented as *x*_*i*,*j*_, representing the position of the *i*-th sparrow in the *j*-th dimension, where *i*=1,2,3,…, *n*, *j*=1,2,…, *d*. The fitness value can be expressed as *F*_*x*_*i*__=*f*([*x*_*i*1_, *x*_*i*2_ ⋯ *x*_*i*  *d*_]).

In each iteration, sparrows with high fitness values, representing about 10% to 20% of the population, are selected as producers. The formula for producer update location can be described using the following equation:

(1) $$\begin{array}{c} X_{i,j}^{t+1}=\left\{\begin{array}{cc} X_{i,j}^{t}\cdot \;\exp\left(\frac{-i}{\alpha \cdot T}\right), & R_{2}<\text{ST},\\ X_{i,j}^{t}+Q\cdot L, & R_{2}\geq \text{ST}. \end{array}\right) \end{array}$$

Among them, *t* indicates the current iteration number. *α*(*α* ∈ (0,1]) is a uniform random number. *T* represents the maximal number of iterations. *Q* denotes a standard normally distributed random number. *L* indicates a matrix of size 1 × *d*, and all elements are assigned to 1. *R*_2_ is the alarm value in the range [0,1]. The range of the safety threshold is [0.5, 1], denoted by ST. When *R*_2_ < ST, it indicates that the predator is not present in the environment and the producer can conduct a large-scale search. When *R*_2_ ≥ ST, it implies that the monitor has detected the predator and the population required to move to a safe place after receiving the alarm signal. Scroungers obtain food by following or competing with producers. The formula for scrounger update location can be described as follows:

(2) $$\begin{array}{c} X_{i,j}^{t+1}=\left\{\begin{array}{cc} Q\cdot \;\exp\left(\frac{X_{worst}^{t}-X_{i,j}^{t}}{i^{2}}\right), & i>\frac{n}{2},\\ X_{p}^{t+1}+\left|X_{i,j}^{t}-X_{p}^{t+1}\right|\cdot A^{+}\cdot L, & i\leq \frac{n}{2}, \end{array}\right) \end{array}$$

where *X*_*p*_ represents the optimal position for the producer. *X*_worst_ represents the global worst position at the current moment. *A* denotes a 1 × *d* matrix, where the elements are randomly assigned to 1 or −1, and the matrix satisfies the equation *A*^+^=*A*^*T*^(*AA*^*T*^)^−1^. When *i* > (*n*/2), it implies that the *i*-th scrounger is in a hungry state with poor fitness and low energy. To increase their energy, scroungers must move to other areas searching for food. When *i* > (*n*/2), the scrounger follows the best-positioned producer to forage.

About 10 to 20 percent of the individuals in the population will perform as monitors. Monitors provide scouting for groups and warn other sparrows to counter predation when danger occurs. The method of updating the monitor position is as follows:

(3) $$\begin{array}{c} X_{i,j}^{t+1}=\left\{\begin{array}{cc} X_{\text{best}}^{t}+\beta \cdot \left|X_{i,j}^{t}-X_{\text{best}}^{t}\right|, & f_{i}>f_{g},\\ X_{i,j}^{t}+K\cdot \left(\frac{\left|X_{i,j}^{t}-X_{\text{worst}}^{t}\right|}{\left(f_{i}-f_{w}\right)+\varepsilon }\right), & f_{i}=f_{g}. \end{array}\right) \end{array}$$

Among them, *X*_best_ indicates the best position in the whole area. *β* denotes a standard normally distributed random number. *K* denotes a random number between [−1,1]. Both *β* and *K* represent the step size control parameter. *f*_*i*_ expresses the present fitness value of the sparrow. *f*_*g*_ and *f*_*w*_ represent the fitness values of the best and worst positions in the whole region, respectively. *ε* is an extremely small constant to prevent the error of zero division. When *f*_*i*_ > *f*_*g*_, the individual is at the border of the population and easily becomes a target of predators. When *f*_*i*_=*f*_*g*_, the sparrow perceives the risk and needs to approach other fellows to ensure safety.

### 3.2. Long Short-Term Memory Network

LSTM is a variant of RNN that overcomes the problem of long-term dependency in RNN. The LSTM consists of input gates, output gates, forgetting gates, and memory cells. The cell unit holds the status information of the present time, which contains the status information of the last time step and the temporary status information of the present time step. When data enter the LSTM network, three gates determine the information that needs to be remembered and forgotten at each time step. The subtle gate control of LSTM brings the addition operation into the network, which improves the gradient disappearance problem to some extent.  Figure 1 illustrates the structure of a single neuron in LSTM.

The output *h*_*t*_ of the LSTM at the moment *t* can be expressed as

(4) $$\begin{array}{c} h_{t}=o_{t}\cdot \;\tanh\left(C_{t}\right), \end{array}$$

where the computation of *o*_*t*_ and *C*_*t*_ can be indicated using the following equations, respectively:

(5) $$\begin{array}{c} o_{t}=\sigma \left(w_{o}\cdot \left[h_{t-1},x_{t}\right]+b_{o}\right), \end{array}$$

(6) $$\begin{array}{c} C_{t}=f_{t}\cdot C_{t-1}+i_{t}\cdot {\tilde{C}}_{t}. \end{array}$$

The calculation methods of *f*_*t*_, *i*_*t*_, and ${\tilde{C}}_{t}$ are as follows:

(7) $$\begin{array}{c} f_{t}=\sigma \left(w_{f}\cdot \left[h_{t-1},x_{t}\right]+b_{f}\right),\\ i_{t}=\sigma \left(w_{i}\cdot \left[h_{t-1},x_{t}\right]+b_{i}\right),\\ {\tilde{C}}_{t}=\tanh\left(w_{c}\cdot \left[h_{t-1},x_{t}\right]+b_{c}\right), \end{array}$$

where *i*_*t*_, *f*_*t*_, and *o*_*t*_ correspond to the input gate, forgetting gate, and output gate, respectively. These gates are functions of the input feature *x*_*t*_ at the current time and the short-term memory *h*_*t*−1_ at the last time. *w*_*i*_, *w*_*f*_, and *w*_*o*_ denote the parameter matrices to be trained, while *b*_*i*_, *b*_*f*_, and *b*_*o*_ represent the bias terms to be trained. *σ* is a shorthand for *sigmoid*, which means the activation function. *C*_*t*_ denotes the neuron state, which indicates long-term memory. *h*_*t*_ is the output of the neuron, which represents the short-term memory. ${\tilde{C}}_{t}$ is the candidate vector, meaning the new knowledge that will be stored in the cell unit.

The activation functions used by the gating structure in the neural unit of LSTM are sigmoid and tan*h*. The definition of the sigmoid activation function is shown as follows:

(8) $$\begin{array}{c} f\left(x\right)=\frac{1}{1+e^{-x}}. \end{array}$$

The calculation method of tan*h* is shown in equation (9).

(9) $$\begin{array}{c} f\left(x\right)=\frac{1-e^{-2x}}{1+e^{-2x}}. \end{array}$$

The output of the sigmoid function is between 0 and 1, which conforms to the physical meaning of the LSTM gating unit. The changes in output and input are positively correlated, which ensures the switching function of the gate control unit. The tanh function causes the output of ${\tilde{C}}_{t}$ to be between [0,1], which is consistent with the center of the feature distribution being 0 in most cases.

LSTM inherits most of the features of RNN while alleviating the problem of gradient disappearance, so it is more suitable for complex financial time series. This paper chooses LSTM as the base model and applies it to stock price trend prediction.

### 3.3. SSA-LSTM Model

The SSA presents the advantages of rapid convergence and excellent search accuracy in optimization problems. Recently, several studies [24–26] have applied an SSA to different engineering fields with good results, which also have practical assistance for our research. Compared with the model in the research [24], we concentrated on optimizing the hyperparameters of the network model for the purpose of minimizing the human influence on the network model and improving the prediction capability of the model. Therefore, we set the learning rate, the time step, the number of neurons in the LSTM layer, the number of neurons in the dense layer, and the epoch number as the target optimization parameters. In this study, the SSA was applied to optimize these target parameters of LSTM to achieve the matching of data features and model structure. The SSA can find the optimal values of LSTM network parameters quickly and efficiently, which enhances the interpretability of the network structure.

#### 3.3.1. Structure of SSA-LSTM

The network architecture of SSA-LSTM mainly consists of an input layer, an LSTM layer, a dense layer, and an output layer. We take the learning rate, epoch number, neuron numbers in the two hidden layers, and time step as the parameter objectives to be optimized by the SSA. The location information of the population and related parameters are randomly initialized after setting the value range of the parameters. In the learning model, we choose to use the “mean squared error (MSE)” as the loss function of LSTM and the fitness function of the SSA. We compute and rank the fitness values in the expectation of finding a set of parameters that minimizes the LSTM error. The formula for the fitness function can be expressed as follows:

(10) $$\begin{array}{c} f=\frac{1}{n}\sum_{1}^{n}{\left({\hat{y}}_{i}-y_{i}\right)}^{2}. \end{array}$$

Among them, *n* is the sample size of the validation dataset. *y*_*i*_ denotes the actual value, and ${\hat{y}}_{i}$ represents the predicted value.

We update the location information of all kinds of individuals by formulas (1)–(3). The optimal value of the target parameter is output when the optimization process satisfies the convergence condition. Otherwise, it will repeat the process of dividing the population, updating the location information, comparing the optimal solution, and updating the fitness value until satisfying the convergence conditions. Finally, we establish the SSA-LSTM model with the structure shown in Figure 2 for stock prediction.

#### 3.3.2. Steps of the SSA

The flowchart is shown in Figure 3. The specific procedure of the SSA to optimize the parameters of the LSTM network can be formulated in six steps as follows:

**Step 1 .**

Preprocessing. The data preprocessing consists of multiple sections: determining input features, data normalization, sorting, and normalization processing. After completing these tasks, we divide the training set and test set proportionally.

**Step 2 .**

Population settings. Set the number of populations, alarm value, number of algorithm iterations, etc. Then, calculate the number of discoverers and monitors from the specified percentage.

**Step 3 .**

Parameter initialization. Generating the search space and initializing the population according to the number of sparrows and target parameters (learning rate, epochs, neuron numbers in the two hidden layers, and time step).

**Step 4 .**

Calculate the fitness value. We use MSE as the fitness function to discover the best and worst individuals by their fitness values.

**Step 5 .**

Location update. The positions of the producer, the predator, and the monitor are updated by formulas (1)–(3). Then, compare the current global optimal solution and adjust the optimal fitness value.

**Step 6 .**

Determine the loop situation. If the optimal fitness value is stabilized or the iteration is completed, output the best value; else, return to Step 4.

The SSA-LSTM model we finally build is based on the algorithm-optimized parameters, which determine the structure of the model and give a final decision-making ability to the model. The process of algorithmic optimization search demonstrates the origin of our parameter settings and model building while maximizing the elimination of human factors and enhancing the interpretability of the model structure and parameters.

## 4. Experiments

This paper uses the Shanghai Composite Index dataset from January 2010 to September 2021, including 2850 days of historical transaction data. The basic stock trading data such as open price and close price are obtained through the Tushare platform. With these trading data, the values of stock technical indicators such as moving average convergence and divergence (MACD) can be calculated by the TA-Lib technical analysis library. In this study, the input features consist of open price, high price, low price, close price, volume, turnover, and MACD. Gaps in the dataset that may arise due to the trade suspension and other reasons need to be removed before the experiment.

We had to validate the prediction effectiveness of different models while using SSA-LSTM models for stock prediction experiments. We employed five models (BP, RNN, LSTM, GRU, and PSO-LSTM) for our comparison experiments. BP is one of the early models used for stock prediction and is the most typical neural network. These two points are the reasons why we choose the BP neural network as the comparison model. RNN is applied in the field of stock prediction due to its obvious advantages in dealing with time-series problems. The LSTM neural network has a more powerful feature extraction ability and generalization ability after solving the shortcomings of RNN, and GRU is another variant of the LSTM model. Considering that our proposed SSA-LSTM model is built based on LSTM and all these models are widely used in stock prediction, we choose BP, RNN, and GRU as part of the comparison experiments. In addition, we reproduce the experiments of using the PSO algorithm to optimize the LSTM model as a way to fully demonstrate the effectiveness of the SSA-LSTM model.

We take 80% of the dataset as the training set for the comparison model and the remaining 20% as the test set. For the PSO-LSTM and SSA-LSTM models, the first 80% of the dataset is used for the optimization algorithm to search for the optimal parameters and train the model, and the last 20% is considered as the test set to test the model generalization error.

The experimental environment is TensorFlow deep learning framework running under Windows, configured with NVIDIA CUDA 10.1 and cuDNN 7.6 deep learning library to accelerate GPU computation; Python version is 3.7, and TensorFlow version is 2.1.

### 4.1. Judgment Criteria

In this paper, we use the mean absolute percent error (MAPE), root mean squared error (RMSE), mean absolute error (MAE), and coefficient of determination (*R*^2^) as the evaluation indicators of the model prediction results. Their formulas are shown as follows:

(11) $$\begin{array}{c} e_{\text{MAPE}}=\frac{1}{n}\sum_{1}^{n}\frac{\left|{\hat{y}}_{i}-y_{i}\right|}{y_{i}},\\ e_{\text{RMSE}}=\sqrt{\frac{1}{n}\sum_{1}^{n}{\left({\hat{y}}_{i}-y_{i}\right)}^{2}},\\ e_{\text{MAE}}=\frac{1}{n}\sum_{1}^{n}\left|{\hat{y}}_{i}-y_{i}\right|,\\ R^{2}=\frac{\sum_{1}^{n}{\left({\hat{y}}_{i}-\bar{y}\right)}^{2}}{\sum_{1}^{n}{\left(y_{i}-\bar{y}\right)}^{2}}. \end{array}$$

Among them, the actual and forecasted values of stock prices are expressed as *y*_*i*_ and ${\hat{y}}_{i}$, respectively. *n* is the sample size of the test dataset.

### 4.2. Optimizing Network Parameters by the SSA

In order to update the network weights more efficiently, Adam was chosen as the optimizer. The dropout is adjusted to 0.1 to prevent overfitting. The number of sparrow populations is set to 10, and the percentage of discoverers is set to 20%. There are five hyperparameters of LSTM that need to be optimized, which are the learning rate, epochs, neuron numbers in the two hidden layers, and the time step. With the basic parameter settings, the search range is initialized to a 10 × 5 matrix. The SSA aims to find the optimal combination of hyperparameters by searching the search space and minimizing the loss on the test set.

We need to set a reasonable search range for the parameters to avoid problems that may occur during the search process, such as a large search range that leads to high consumption of resources. We analyzed some research papers [27–29] based on LSTM models for forecasting the Chinese stock market and some literature mentioned in related works. The parameter values set in these studies were heavily adjusted and tested, and the experimental results all met the researchers' expectations. Therefore, the parameter values set in these studies have some reference value for us to set the search range of the parameters. We found that the learning rates set by most of the researchers were between 0.001 and 0.01, and there were few learning rates less than 0.001 or higher than 0.01. Most of these studies that illustrate the parameter settings keep the number of hidden layer neurons less than 100 and the time step less than 20. In addition, many studies set the epoch within 100 or around 200, and fewer studies chose a higher number of epochs. Given the analysis of these related studies, we set the appropriate parameter search range: the learning rate is defined between [0.001, 0.01], the number of neurons in both the LSTM and DENSE layers is between [1, 100], and the time step is between [1, 20]. We have tested and found that epochs larger than 100 hardly bring any changes to our experiments, and considering the pressure of the experimental environment, we finally set the search range of epochs at [10, 100].

With the search range of the target optimization parameters, we will obtain the optimal parameters by the SSA.  Figure 4 and Table 1 show the optimization process for each parameter.

The analysis shows that the fitness value of the algorithm reaches a minimum at the third iteration and keeps the minimum value constant thereafter. Meanwhile, the values of each target parameter also remain stable after the third iteration, indicating that the SSA has found the optimal parameters of the model. We can clearly observe the changes in the target parameters during the optimization process in Table 1. After the third iteration, the fitness value remains unchanged at the minimum value of 0.31894529, and the other parameters also remain constant after reaching the optimal values.

From Table 2, the optimal parameters of LSTM obtained by the SSA are the learning rate of 0.00616353, the epoch of 90, 33 neurons of the LSTM layer, 79 neurons of the dense layer, and the time step of 5. We construct a prediction model for stock forecasting based on the optimal values of the parameters obtained by the SSA optimization.

### 4.3. Experimental Results and Analysis

This part analyzes the capability of SSA-LSTM for price trend prediction. Classical models such as BP, RNN, LSTM, and GRU are widely used in the field of stock prediction. We use these stock prediction models as the comparison models of SSA-LSTM for experiments, which can directly test the effectiveness of the model proposed in this paper. In addition, we also reproduce the PSO algorithm for optimizing the LSTM model and use PSO-LSTM as a comparison model in this paper. Based on testing the predictive ability of SSA-LSTM, we can further compare the effectiveness of two swarm intelligence algorithms, SSA and PSO, for optimizing LSTM models.

Figure 5 illustrates the forecasting results of BP, RNN, LSTM, GRU, PSO-LSTM, and SSA-LSTM. The parameter search range of the PSO algorithm-optimized LSTM model is consistent with that in Table 2, and the final optimal hyperparameter results are as follows: the learning rate is 0.00729531, the number of model training is 87, the number of neurons in the first and second hidden layers is 76 and 57, and the time step is 10. We establish the prediction model with the optimal parameters found by PSO for experiments, and the prediction outcome is presented in Figure 5(e).

From Figure 5(a), we can clearly observe that the classical BP network can roughly predict the stock trend. However, we found that BP has poor prediction performance when the stock price fluctuates drastically, and there is a significant error between the prediction curve and the actual curve. The RNN model, which is good at dealing with time-series problems, performs better forecasting ability than BP. From Figure 5(b), we can notice that the trend of the RNN prediction curve is roughly similar to the actual curve. However, there is still a significant lag in the prediction of RNN, and there is a relatively large error at certain inflection points. As a powerful model for the time-series problem, the LSTM network solved the gradient vanishing problem of RNN. It is obvious from the prediction curves that the prediction performance of LSTM has been improved and the error of prediction results has been reduced. As another improved model of LSTM, GRU has further diminished the lag in prediction and holds a higher prediction accuracy. Although the fitting capability of GRU has shown a significant improvement compared with that of LSTM, the prediction at the inflection point is still unsatisfactory. After applying the swarm intelligence optimization algorithm to optimize the model parameters, we have discovered that the optimized model provides a better generalization and fitting ability. The excellent forecasting performance of the PSO-LSTM model confirms the effectiveness of the PSO algorithm. It is not difficult to observe that the prediction curve of the SSA-LSTM model is closest to the actual curve by comparing it with other prediction models. The minor deviations between the predicted and actual values and the minor errors at the prediction inflection points indicate that the SSA-LSTM model performs a better fit ability than other forecasting methods. Given the analysis of the prediction curves, we can observe that the SSA-LSTM model outperforms other prediction models in prediction accuracy and reduction of prediction lags.

To facilitate a more intuitive and accurate comparison of prediction effects between the models and to reflect the performance advantages of the SSA-LSTM model, the results of the evaluation indexes of each model are presented in Table 3.

As shown in Table 3, BP is an earlier model applied to stock forecasting, and its four evaluation indexes have values of 0.0347, 147.7001, 116.8226, and 0.6956. The relatively high values of MAPE, RMSE, and MAE represent the more obvious prediction error of BP, while the smaller *R*^2^ indicates the weaker fitting ability of BP. The prediction ability of RNN has improved significantly compared with BP, and the values of MAPE, RMSE, MAE, and *R*^2^ are 0.0175, 74.9063, 58.4909, and 0.9217, respectively. From the prediction curves and evaluation metrics, the prediction of RNN is still not accurate enough. The LSTM model is the most classical method in the field of stock prediction, and its evaluation metrics show that the prediction ability has been enhanced significantly after solving the gradient vanishing problem of RNN. The index values of LSTM are 0.0115, 49.7854, 37.6467, and 0.9663, which still have more errors compared with the model proposed in this paper. GRU is an optimization model based on LSTM. We can observe from the experimental results that the values of MAPE, RMSE, MAE, and *R*^2^ of GRU are 0.0115, 49.7854, 37.6467, and 0.9663, which indicate that the indicators of error are lower than LSTM and the values of coefficient of determination are slightly higher than LSTM. The prediction ability of the model has improved substantially after applying the swarm intelligence algorithm to optimize the LSTM. The prediction evaluation index values of the PSO-LSTM model are 0.0097, 43.0891, 31.9715, and 0.9741, which are significantly better than the classical prediction methods and illustrate the effectiveness of the swarm intelligence algorithm for optimizing the LSTM model parameters. The SSA-LSTM model proposed in this paper uses a novel SSA to optimize the LSTM, and its prediction results are further improved compared with the PSO-LSTM as expected. The values of MAPE, RMSE, and MAE corresponding to the SSA-LSTM model are 0.0093, 41.9505, and 30.5300, respectively. The MAPE of the SSA-LSTM model was 73.2%, 46.9%, 27.9%, 19.1%, and 4.1% lower than that of the BP, RNN, LSTM, GRU, and PSO-LSTM models, respectively; the RMSE was reduced by 71.6%, 44.0%, 24.8%, 15.7%, and 2.6% compared with that of the other five models, respectively; and the MAE indicator was decreased by 73.9%, 52.2%, 27.7%, 18.9%, and 4.5% compared with that of the other five models, respectively. The cases of all three metrics indicate that the error between the forecasted and actual values of SSA-LSTM is smaller and the prediction accuracy is higher than that of other models. The *R*^2^ of SSA-LSTM is the closest to 1 among all models in Table 3, which denotes that the model possesses a stronger fitting ability. All the experimental results illustrate that the SSA-LSTM model has the best prediction ability and prediction effect relative to other methods.

According to the above analysis, the SSA-LSTM model is more effective and has higher forecasting accuracy than the traditional network model when dealing with stock time-series data.

## 5. Conclusion

We proposed an SSA-LSTM model for stock trend prediction in response to the problem that the selection of hyperparameters in LSTM networks was often based on subjective experience and existing research. The parameters of the LSTM model are optimized by the sparrow search algorithm, which objectively explains the origin of the model network structure and parameter settings. This process minimizes the influence of human factors on the stock prediction process and improves the generalization ability and prediction effect of the model. This paper selected the representative Shanghai Composite Index dataset in the Chinese financial market for training and testing the model. The experiments are compared with the PSO-LSTM model and some other classical machine-learning methods, and the results prove that the SSA-LSTM model possesses high prediction accuracy for stock price trend prediction. In addition, the reliability and adaptability of the SSA-LSTM model to the Chinese stock market are also verified.

With the complex financial market, the SSA-LSTM model can rapidly and accurately grasp the data characteristics and achieve high-precision price trend prediction, which can reduce the risk to investors to a certain extent. This model has the capability to handle time-series data efficiently and also has a certain application value for other time-series problems.

## Figures and Tables

**Figure 1:** Neural unit structure of LSTM.

**Figure 2:** SSA-LSTM model architecture.

**Figure 3:** Flowchart of the SSA.

**Figure 4:** Optimization iterative process of SSA-LSTM.

**Figure 5:** Comparison between prediction results of each model.

**Table 1:** Optimization iterative process of SSA-LSTM.

Algorithm iterations	Learning rate	Epoch	Neuron numbers in the first hidden layer	Neuron numbers in the second hidden layer	Time step	Fitness value
1	0.00666221	96	76	46	13	0.67514376
2	0.00666527	97	32	78	4	0.50569965
3	0.00616353	98	33	79	5	0.31894529
4	0.00616353	98	33	79	5	0.31894529
5	0.00616353	98	33	79	5	0.31894529

**Table 2:** Results of hyperparametric optimization.

Parameter	Search range	Optimal value
Learning rate	[0.001, 0.01]	0.00616353
Epoch	[10, 100]	98
Neuron numbers in the first hidden layer	[1, 100]	33
Neuron numbers in the second hidden layer	[1, 100]	79
Time step	[1, 20]	5

**Table 3:** Evaluation results of models.

Model	MAPE	RMSE	MAE	*R* ^2^
BP	0.0347	147.7001	116.8226	0.6956
RNN	0.0175	74.9063	58.4909	0.9217
LSTM	0.0129	55.7954	42.2065	0.9566
GRU	0.0115	49.7854	37.6467	0.9663
PSO-LSTM	0.0097	43.0891	31.9715	0.9741
SSA-LSTM	0.0093	41.9505	30.5300	0.9754

## Data Availability

Data are available from the following link: https://tushare.pro/.
